# Moxibustion Modulates Sympathoexcitatory Cardiovascular Reflex Responses Through Paraventricular Nucleus

This article has been retracted.

**DOI:** 10.3389/fnins.2018.01057

**Published:** 2019-01-21

**Authors:** Ling Cheng, Peng Li, Yash Patel, Yiwei Gong, Zhi-Ling Guo, Huangan Wu, Shaista Malik, Stephanie C. Tjen-A-Looi

**Affiliations:** ^1^Eastern Hospital Affiliated to Tongji University, Shanghai, China; ^2^Susan Samueli Integrative Health Institute, University of California, Irvine, Irvine, CA, United States; ^3^Shanghai Research Institute of Acupuncture and Meridian, Shanghai University of Traditional Chinese Medicine, Shanghai, China

**Keywords:** gastric distention, deep peroneal nerve, acupoint specific, paraventricular nucleus, sympathoexcitatory cardiovascular reflex response

## Abstract

Electroacupuncture (EA) point specific (ST36-37) stimulation decreases cardiovascular reflex responses through supraspinal regions such as the hypothalamic paraventricular nucleus (PVN) while mechanical stimulation of acupoints decreases pressor responses through peripheral thermal transient receptor potential vanilloid type-1 (TRPV1). Moxibustion generating heat applied at acupoint in combination with antihypertensive drugs decreases elevated blood pressure. We hypothesized that moxibustion modulates sympathoexcitatory cardiovascular responses through the hypothalamic PVN and peripheral heat sensitive TRPV1 in the absence of antihypertensive drugs. Rats were anesthetized, ventilated, and heart rate and mean blood pressure were monitored. Gastric distention induced consistent pressor reflex responses every 10-min. Thirty-minutes of bilateral moxibustion at the acupoint ST36, overlying the deep peroneal nerves, reduced the gastric distention evoked elevation in blood pressure. Blood pressure reflex responses were not reduced by both EA and moxibustion at G39. The moxibustion inhibition but not EA inhibition of the cardiovascular responses was reversed with blockade of local heat sensitive TRPV1 at ST36. Accordingly, activation of thermal TRPV1 by moxibustion at an average of 44.2°C in contrast to 40°C reduced the pressor responses. Naloxone, an opioid receptor antagonist, microinjected into PVN inhibited transiently the effect of moxibustion. Thus, activation of peripheral heat sensitive TRPV1 mediated the moxibustion-inhibition, but not EA-inhibition, of sympathoexcitatory cardiovascular reflex responses through hypothalamic PVN opioid system.

## Introduction

Moxibustion has been used to treat gastrointestinal problems such as irritable bowel syndrome (Liu et al., 2015; Shi et al., 2015) but not much is known about its effect on hypertension. Few clinical studies indicate that moxibustion in the presence of antihypertensive drugs may reduce hypertension, but the efficacy and mechanisms underlying moxibustion in the absence of drugs are unknown (Xiong et al., 2014; Lee et al., 2016). We have shown in a series of studies in men and animals that electroacupuncture (EA) at specific acupoints activating peripheral nerves modifies sustained hypertension and reflex elevated blood pressure through reduction of sympathetic activity (Chao et al., 1999; Tjen-A-Looi et al., 2004; Li et al., 2004, 2016; Crisostomo et al., 2005). In this respect, specific central regions and neurotransmitter systems in the hypothalamus and medulla participate in the central processing of the action of acupuncture (Chao et al., 1999; Crisostomo et al., 2005; Li et al., 2009, 2010, 2015; Tjen-A-Looi et al., 2009; Moazzami et al., 2010; Tjen-A-Looi et al., 2013). The current study investigates in the absence of antihypertensive drugs the effect as well as underlying mechanisms of moxibustion at specific acupoint on sympathoexcitatory cardiovascular reflex responses in rats.

Cardiovascular regions in the central nervous system (CNS) such as rostral ventrolateral medulla (rVLM), and paraventricular nucleus (PVN) are activated during stimulation of visceral spinal afferents that leads to increases in blood pressure (Tjen-A-Looi et al., 2003, 2016). A series of studies have shown that through actions in rVLM stimulation of both gallbladder and gastric afferent activates splanchnic nerve and increases blood pressure (Li et al., 2002, 2010; Tjen-A-Looi et al., 2004; Crisostomo et al., 2005; Zhou et al., 2005a; Tjen-A-Looi et al., 2006; Moazzami et al., 2010). The PVN projects directly to the rVLM and to a lesser extent to the intermediolateral column of the spinal cord (Pyner and Coote, 1999; Hardy, 2001; Pan, 2004; Chen and Toney, 2010) and contributes to the descending neuronal pathway regulating sympathetic outflow in the rVLM (Tjen-A-Looi et al., 2016). In particular, the parvocellular PVN is critical in regulation of sympathoexcitatory cardiovascular pressor reflex responses such as during activation of splanchnic and cardiac sensory fibers (Xu et al., 2012; Tjen-A-Looi et al., 2016).

Manual acupuncture (MA) and EA modulate pressor responses that are induced by chemical, mechanical, or electrical stimulation of visceral afferent nerves (Li et al., 1998, 2001, 2002; Chao et al., 1999; Tjen-A-Looi et al., 2003, 2004; Crisostomo et al., 2005; Zhou et al., 2005a,b). We observe that EA at P5-6 decreases ischemic myocardial dysfunction (Chao et al., 1999) through decrease of oxygen demand demonstrating that acupuncture reduces demand-induced myocardial ischemia and blunts the sympathoexcitatory reflex elevation of blood pressure (Li et al., 1998). EA stimulation at P5-6 or ST36-37 activating respectively median or deep peroneal nerves and reducing elevated sympathetic activity decreases cardiovascular reflex vasoconstriction and elevation in blood pressure (Li et al., 1998, 2002; Chao et al., 1999; Tjen-A-Looi et al., 2004). With this regard, sympathoexcitatory cardiovascular responses are decreased by EA stimulation at both P5-6 and ST36-376. In addition, sympathetic premotor cardiovascular rVLM cells important for sympathetic outflow participate in central processing of the actions of EA and MA (Tjen-A-Looi et al., 2003, 2004; Zhou et al., 2005b). Recently, we demonstrate that EA-modulation of visceral induced excitatory cardiovascular responses also involves the hypothalamic PVN (Tjen-A-Looi et al., 2016). We showed that the rVLM-projecting PVN neurons important in regulation of cardiovascular responses participate in central processing of the modulatory actions of EA (Tjen-A-Looi et al., 2016). Thus, parvocellular PVN appears to be an important cardiovascular region in the hypothalamus that processes cardiovascular reflex responses and contributes to the actions of acupuncture.

Moxibustion, like EA and MA, is a form of acupoint stimulation. The acupoints are stimulated with heat generated by moxibustion (Wang et al., 2013). Moxibustion at specific acupoints relieves pain and modulates gastric motility and irritable bowel syndrome (Su et al., 2014; Liu et al., 2016; Zhao et al., 2016). Moxibustion applied at acupoint ST36 modulated gastric motility in rats (Su et al., 2014) suggesting that activation of peripheral nerves underlying the acupoint modulates gastrointestinal responses (Tjen and Fu, 2017). Moreover, stimulation of acupoints with either EA or MA modulates elevated blood pressure (Tjen-A-Looi et al., 2004; Zhou et al., 2005b) but through different peripheral mechanisms (Guo et al., 2018). In this regard in contrast to EA, peripheral transient receptor potential vanilloid type-1 (TRPV1) at acupoint P6 contributes to the effect of MA (Guo et al., 2018) suggesting differential underlying mechanisms are involved during stimulation of acupoints. The TRPV1 polymodal receptor is activated by heat greater than 42°C, mechanical stimuli, during EA in analgesia at ST36, and others (Tominaga et al., 2001; Birder et al., 2002; Pan and Chen, 2004; Nakagawa and Hiura, 2006; Caterina, 2007; Xin et al., 2016). Although activation of mechanosensitive TRPV1 during MA at P6 reduces elevated blood pressure, no information is available on the role of thermosensitive TRPV1 at acupoint ST36 during EA or moxibustion on sympathoexcitatory cardiovascular reflex responses. We hypothesize that moxibustion activating peripheral thermal-sensitive TRPV1 at acupoint ST36 decreases reflex hypertension through the opioid system in the PVN. A preliminary report of this work has been presented (Gong et al., 2018).

## Materials and Methods

### Surgical Procedures

Experimental preparations and protocols were reviewed and approved by the Institutional Animal Care and Use Committee of the University of California, Irvine, CA, United States. The study conformed to the American Physiological Society “Guiding Principles for Research Involving Animals and Human Beings.” The minimal possible number of rats was used to obtain reproducible and statistically significant results. Studies were performed on adult Sprague-Dawley male rats (400–600 g). Rats were anesthetized with ketamine (100 mg/kg im) and anesthesia was maintained with αα-chloralose (5 mg/kg iv). Additional doses of α-chloralose were given as necessary to maintain an adequate level of anesthesia, as determined by the lack of response to noxious toe pinch and corneal reflex, and the ability to artificially maintain a consistent respiratory rate. The trachea was intubated for artificial respiration using a ventilator (Model 661, Harvard Apparatus). The respiration was maintained with room air enriched with oxygen. The right jugular vein was cannulated for administration of fluids. The right or left carotid artery was cannulated and attached to a pressure transducer (P23XL, Ohmeda) to monitor arterial blood pressure. Heart rate was derived from the pulsatile blood pressure pulse using a biotech Gould Instrument (Cleveland, OH, United States). Blood pressures and heart rates were recorded and analyzed offline with a computer and CED Spike 2 Windows software. Throughout the experiment arterial blood gases and pH were measured periodically with a blood gas analyzer (ABL5, Radiometer America) and were kept within normal physiological limits (PCO_2_ 35–40 mmHg, and PO_2_ 100–150 mmHg) by adjusting ventilatory rate or volume and enriching the inspired O_2_ supply. Arterial pH was maintained between 7.35–7.45 by infusion of 8% sodium bicarbonate. Body temperature was kept between 36° and 38°C with a heating pad and an external heat lamp. Fur was removed in the region of the ST 36 or G39 acupoint located bilaterally on the hind limbs.

To stimulate gastric afferent by gastric distention, a 2-cm diameter unstressed dimension latex balloon attached to a polyurethane tube (3 mm diameter) was inserted into the stomach through the mouth and esophagus (Tjen-A-Looi et al., 2009). During insertion and passage through the esophagus, the balloon was palpated manually to confirm positioning of the balloon inside the stomach. A syringe was attached to the cannula to inflate and deflate the balloon with air, while a manometer through a T-connection was used to monitor balloon pressure. Transmural pressure was determined by measuring the pressure required to inflate the balloon with the various volumes of air before it was inserted into the stomach (Li et al., 2002). Distention pressures were selected to fall within the range that a rat normally experiences during ingestion of food and fluids in a single meal (Davison and Grundy, 1978; Baird et al., 2001). The balloon was deflated within 30 s after reaching the maximum increase in blood pressure. The positioning of the balloon was verified post mortem to be in the stomach.

To investigate the action of moxibustion in the hypothalamus, the animal was stabilized with a Kopf stereotaxic head frame. A craniotomy was performed to expose the dorsal surface of the cortex and gain access to the PVN. An injection cannula and microsyringe (Hamilton) fixed to a microinjection probe with inner diameter of 0.4 mm was inserted into the PVN to deliver antagonist, vehicle control or Chicago blue dye. Using visual approximation, the microinjection probe was positioned perpendicularly to the dorsal surface of the cortex 1.8 mm posterior to the Bregma, 0.5 mm lateral to the midline, and advanced ventrally 7.5–7.8 mm to reach the PVN. These coordinates provide access to a region that has been found by others to contain sympathetic related cells (Kenney et al., 2003; Chen and Toney, 2010; Cardoso et al., 2012). At the end of experiment, the microinjection site was marked with Chicago blue dye for later histological confirmation following delivery of drugs into the PVN.

### Stimulating Methods

Gastric distensions were repeated 10 times to establish consistent pressor responses. Recovery of at least 10 min between gastric distensions prevented tachyphylaxis of the cardiovascular responses. To examine effects of moxibustion, acupoint ST36 (the anterolateral side of the hind-limb near the anterior crest of the tibia below the knee, under the tibialis anterior muscle that overlies the deep peroneal nerves) was stimulated with moxibustion for 30 min during three gastric distensions following two initial consistent pressor responses. Additional five pressor responses were evaluated after cessation of thermal stimulation to determine long-lasting effect of thermal stimulation at ST36. Total of 10 gastric distention induced pressor responses were evaluated. To examine the point specific thermal-sensitive effect, acupoint G39 (above the ankle at the lower one third of the hind limb overlying superficial peroneal nerves) also was stimulated similarly with heat generated by moxibustion. Responsiveness to specific temperature was evaluated with moxibustion–induced heat at 1 or 2 cm distance from the surface of the hind limbs at acupoint ST36 or G39 (Su et al., 2014). Temperature was measured with probe and thermometer (Fluke 51 II Thermometer) placed on the skin without fur during thermal stimulation at 15 and 30 min. To achieve and maintain the temperatures, the adjustment of the distance from the moxibustion stick to the surface of the skin and the tapping off the ash at end of the stick were performed frequently. Once the temperatures were achieved, the distance was determined and held constant. To determine the similarity of EA and moxibustion on sympathoexcitatory reflex responses, EA at G37-39 and ST36-37 on increases in blood pressure were evaluated in 11 other rats. Needles (40-gauge made by Suzhou Medical Appliance, Suzhou, China) were inserted at ST36-37 at a depth of 3–5 mm and G37-39 at depth of 1–2 mm bilaterally and connected to an isolation unit and stimulator (model S88, Grass, West Warwick, RI) to deliver bipolar stimuli at frequency of 2 Hz, duration of 0.5 ms, and current of 1–4 mA for 30 min. To ensure that twitches by the stimulation of motor fibers (Li et al., 2016) do not contribute to the effects of EA, gallamine triethiodide (4 mg/kg) was administered into the vein after insertion of needles and before the application of EA (Li et al., 2006).

### Methods of Blockade

The role of TRPV1 at acupoint ST36 during action of bilateral moxibustion on gastric distention induced pressor responses was determined with bilateral administration of TRPV1 antagonist iodoresiniferatoxin (Iodo-RTX; 0.1 mM; 10 μl) (Guo et al., 2018). The vehicle control 5% dimethylsulfoxide (DMSO) was administered bilaterally at ST36. The antagonist or vehicle was administered with a hypodermic needle at acupoint ST36 following moxibustion or EA. The proper site and depth of hypodermic needle insertion was confirmed with brief EA stimulation at ST36-37 (placed at a depth of about 3–5 mm) inducing slight repetitive paw twitches in the rats treated with moxibustion. The twitches confirmed stimulation of motor fibers in the mixed deep peroneal nerve bundle (Li et al., 2016). In the hypothalamus, the roles of opioid receptors in the PVN during effect of moxibustion were evaluated by microinjection of the non-specific antagonist naloxone (100 nM, 50-75 nl, Sigma Aldrich, St. Louise, MO, United States) (Tjen-A-Looi et al., 2007) or 0.9% saline vehicle control. An injection cannula and microsyringe (Hamilton) fixed to a pipette were used to administer naloxone or saline into the PVN. Unilateral microinjection allows maintenance of optimal physiological state in studies of EA-modulation of cardiovascular responses (Li et al., 2001; Tjen-A-Looi et al., 2012). With this regard, we investigated the PVN during the effect of heat generating moxibustion on pressor responses with unilateral blockade of opioid receptors.

#### Experimental Protocols

##### 1. Gastric distention evoked reflexes

After the surgical procedures, experiment was conducted following a 30 min stabilization period. Repeated gastric distention was evaluated for consistent increase in blood pressure (Li et al., 2002). After obtaining the maximal cardiovascular pressor response, air was withdrawn from the balloon. Typically, the pressor response was observed within 10 sec following inflation of the balloon. The pressor reflex in mean arterial pressure (MAP) was calculated as the difference in MAP before gastric distention and MAP at the peak of the reflex response. After the completion of each experiment, rats were euthanized with intravenous KCl under deep anesthesia.

##### 2. Moxibustion-inhibition of gastric distention responses

Consistency of increase in blood pressure to gastric distention was evaluated in a group of five animals. Moxibustion-inhibition (ST36) of the increases in MAP was examined in nine other rats. Five of the nine rats were treated with moxibustion 1-cm distance from acupoint ST36 while the other four rats were subjected to the thermal stimulation at 2-cm distance from the skin.

##### 3. Point specific moxibustion-inhibition of pressor responses

Point specific moxibustion-modulation of gastric distention reflex responses was determined by stimulating two different acupoints, including ST36 or G39 at 1-cm distance from the skin. The moxibustion effect at ST36 was evaluated in five rats listed in above protocol (2). In four other animals, eight pressor responses were evaluated during and after 30 min moxibustion at acupoint G39 after obtaining two consistent responses to gastric distension.

##### 4. Electroacupuncture-inhibition of gastric distention responses

Following consistent increases in blood pressure with at least two gastric distentions, cardiovascular reflex responses were measured during 30 min EA at G37-39 (*n* = 5) or EA at ST 36-37 (*n* = 6) in rats. The reflex responses to EA were determined during three gastric distentions. Thereafter, five more gastric distentions were performed every 10 min to evaluate the long lasting inhibitory responses.

##### 5. Thermal sensitive TRPV1 in moxibustion-inhibition and EA-inhibition of pressor responses

Role of TRPV1 during moxibustion-inhibition of the increases in MAP was examined in 12 animals. At ST36 acupoint, TRPV1 was blocked with Iodo-RTX 5 min following termination of moxibustion to evaluate its role in mediating the actions of moxibustion on pressor responses in six of the 12 rats. As a control for the receptor blockade study, DMSO (5%) was injected at the acupoint in six of the 12 subjects tested for ST36 moxibustion-inhibition. In addition, TRPV1 was blocked with Iodo-RTX 5 min following termination of EA ST36-37 to evaluate its role in EA-inhibition of pressor responses in six other rats, listed in protocol (4).

##### 6. Influence of opioid receptor blockade in PVN on moxibustion-inhibition of pressor responses

Role of PVN in moxibustion-inhibition of the increase in MAP was evaluated in eight animals. Two reproducible pre-moxibustion control values were obtained followed by 30 min of moxibustion at the ST36 acupoints. Saline was microinjected into PVN after 20 min of moxibustion. Five min after the end of moxibustion, naloxone was administered into the PVN of five rats. To confirm the role of opioids in moxibustion-inhibition, the effect of naloxone on the pressor responses in the absence of moxibustion was examined in four other animals.

##### 7. Histology

At the end of each experiment, animals were euthanized under deep α-chloralose anesthesia followed by iv injection of saturated KCl. Microinjection sites were marked by microinjection of 2% Chicago blue dye. The brain was removed and fixed in 10% paraformaldehyde for at least 48 hr. Brains were sliced with a microtome cryostat into 40 μm sections. The sites of microinjection were identified and reconstructed with the aid of a microscope (Nikon) and software (Corel presentation) according to the atlas of Paxinos and Watson (2009).

#### Statistical Analysis

Means and standard errors of mean blood pressure and heart rate at rest were compared over time using a repeated-measures analysis of variance (ANOVA) followed by the Student Newman Keuls Test to examine for non-random variation. In the distension-response protocol, comparisons by ANOVA were made between blood pressure responses before and after EA at each increment in gastric volume. Student *t*-test was used to compare responses among groups. The 0.05 probability level was chosen to determine statistical significance.

## Results

### Moxibustion-Inhibition of Gastric Distention Evoked Pressor Responses

Gastric distention increased blood pressure through activation of splanchnic afferent and induced sympathoexcitatory cardiovascular reflex responses (Li et al., 2002). Repeated stimulation of gastric afferent every 10 min displayed consistent increases in MAP during application of 30-min moxibustion 2-cm distance from the skin at acupoint ST36 showing temperatures lower than 40 ± 0.4°C (MAP, Figure 1A). On the other hand, application of 30-min moxibustion 1-cm distance from the skin at acupoint ST36 yielding temperature of 44.2 ± 0.6°C reduced the elevated blood pressure responses for 40 min (Figure 1B). Thus, moxibustion applied with different temperature at acupoint ST36 displayed differential inhibitory outcomes. Baseline blood pressures throughout the experiments were not significantly different. Heart rates also were not altered during the cardiovascular responses.

**FIGURE 1:** Moxibustion inhibition of sympathoexcitatory cardiovascular reflex responses is temperature dependent and acupoint specific. Consistent elevated blood pressure reflex responses (every 10 min) were reduced by moxibustion at ST36 generating heat at temperature between 43 and 46°C **(A)**. Moxibustion temperature between 39 and 41°C did not influence the consistent gastric distention induced pressor responses **(B)**. Moxibustion application at acupoint G39 at temperature between 43 and 46°C also did not reduce the consistent increases in blood pressure **(C)**. Application of EA at ST36-37 also did not reduce the pressor responses **(D)**. Line underneath the histogram bars display the time of duration (30 min) of moxibustion and EA. Numbers below each bar represent the means and SEM of baseline blood pressures. ^∗^ indicates significant different in pressor responses compared with blood pressure increases prior to application of moxibustion or EA.

### Point Specific Moxibustion-Inhibition of Pressor Responses

Consistent gastric distention sympathoexcitatory cardiovascular reflex responses were examined for point specific effects. Moxibustion at average temperature of 44.2 ± 0.6°C applied at ST36 or G39 modulated the reflex responses differentially. Heat stimulation with moxibustion at G39 acupoint did not reduce the pressor responses (Figure 1C) in contrast to ST36 (Figure 1B). Thirty minutes of EA (G37-39) stimulating superficial peroneal nerve also did not reduce the blood pressure reflex responses (Figure 1D) supporting the importance of acupoints ST36 in reducing pressor responses.

### Thermal Sensitive TRPV1 in Moxibustion-Inhibition of Pressor Responses

To determine the peripheral mechanism at acupoint ST36 on the inhibitory effect of moxibustion on sympathoexcitatory cardiovascular responses, the heat sensitive TRPV1 receptor underneath the acupoint was blocked with iodoresiniferatoxin. The TRPV1 blockade transiently reversed the inhibitory effect of moxibustion in contrast to DMSO vehicle (Figures 2A,B). The reversal of moxibustion-inhibition with the TRPV1 antagonist compared with vehicle DMSO on the pressor responses was significantly different (*P* = 0.019).

**FIGURE 2:** Moxibustion inhibits the pressor responses through peripheral TRPV1. Gastric distention (every 10 min) induced increases in blood pressures reduced by moxibustion was reversed transiently following blockade of TRPV1 underneath acupoint. The moxibustion inhibition lasted at least another 20 min after the antagonism **(A)** in contrast to administration of vehicle DMSO **(B)**. Blockade of TRPV1 at ST36 during EA did not reverse the EA-inhibition of the gastric distention induced increases in blood pressure **(C)**. Letters shown in the histogram bars in Panel **A** correspond with the blood pressure tracings a-f. Numbers below each bar represent the means and SEM of baseline blood pressures. ^∗^ indicates significant different in pressor responses compared with blood pressure increases prior to application of moxibustion. # indicates significant reversal of moxibustion-inhibition compared with pressor response immediately before the TRPV1 blockade.

### Thermal Sensitive TRPV1 in EA-Inhibition of Gastric Distention Responses

To examine the peripheral mechanism at acupoint ST36 on the inhibitory effect of EA on sympathoexcitatory cardiovascular responses, the heat sensitive TRPV1 receptor underneath this acupoint was blocked with iodoresiniferatoxin. Our previous study shows that EA ST36-37 reduced the elevated blood pressure responses during repeated gastric distention (Zhou et al., 2005a). Present study showed that the TRPV1 blockade did not reverse the inhibitory effect of EA (Figure 2C). Since DMSO did not affect the inhibition on the cardiovascular reflex responses, DMSO was not re-examined in the presence of EA. In addition, the reversal of moxibustion-inhibition compared with EA-inhibition on the pressor responses following TRPV1 antagonist administration was significantly different (*P* = 0.012) suggesting that the peripheral mechanisms at ST36 in reducing elevated blood pressure are dissimilar.

### Role of Opioids in PVN on Moxibustion-Inhibition of Pressor Responses

To establish participation of the hypothalamus during the moxibustion inhibition on elevated blood pressure responses, opioid receptors were examined in the PVN. Naloxone in contrast to saline in the PVN reversed the moxibustion inhibition on pressor responses (Figure 3).

**FIGURE 3:** Moxibustion inhibits cardiovascular reflex responses through opioids in PVN. Microinjection of naloxone in PVN reversed the moxibustion inhibition on pressor responses induced every 10 min. The moxibustion inhibition lasted at least another 30 min after the opioid receptors blockade. Microinjection of saline did not influence moxibustion inhibition on the gastric distention evoked elevated blood pressures. Numbers below each bar represent the means and SEM of baseline blood pressures. ^∗^ indicates significant different in pressor responses compared with blood pressure increases prior to application of moxibustion. # indicates significant reversal of moxibustion-inhibition compared with pressor response immediately before the TRPV1 blockade.

### Histology

Sites of microinjection marked with Chicago blue dye were confirmed histologically. The sites were determined by the location of microinjection tracks and dye spots. The PVN microinjection sites were confirmed to be 0.4–0.6 mm lateral to the midline and 1.6–1.75 mm from the ventral surface. Data from two microinjections of naloxone that were outside the PVN and did not reverse the effects of moxibustion were not included. Figure 4A displays a coronal section of 60 microns showing the site of microinjection. Figure 4B represents a composite map of all sites closely matched with the rat brain atlas (Paxinos and Watson, 2009).

**FIGURE 4:** Microinjection site marked with an arrow in PVN is displayed in the coronal section **(A)**. Composite map displays the sites of microinjections **(B)**. Coronal sections of the hypothalamus PVN caudal to bregma at 1.8 and 2.1 show the sites with ^∗^. Sites shown with o indicate microinjections outside the PVN.

## Discussion

The present study investigates the effect and underlying mechanisms in the reduction of elevated blood pressure by heat generating moxibustion. The study examined four aspects that are important in the actions of moxibustion inhibition of sympathoexcitatory cardiovascular reflex responses. First, we have observed that the effect of moxibustion is temperature dependent. A temperature greater or at 43°C at the surface of the skin at acupoint ST36 decreases gastric distention induced reflex increases in blood pressure. Secondly, the temperature-dependent moxibustion inhibitory effect on gastric distention induced cardiovascular responses also is related to point specificity. Moxibustion similar to EA applied at ST36, in contrast to G39, significantly decreases the gastric distention induced pressor response (Tjen-A-Looi et al., 2004; Zhou et al., 2005a). As such, previous (Tjen-A-Looi et al., 2004; Zhou et al., 2005a) and current data show that EA and moxibustion share similar point specific modification of pressor responses. Third, blockade of TRPV1 receptor at acupoint ST36 reverses the inhibitory effect of moxibustion. On the other hand, blockade at ST36 is unable to reverse EA-inhibition of reflex elevation of blood pressure. In this respect, heat sensitive receptor TRPV1 activation by moxibustion appears to be important in the inhibition of the pressor response while this receptor activation is not involved during EA-inhibition. Importantly, we demonstrate that the inhibitory effect of moxibustion on cardiovascular reflex responses includes opioid receptor activation in hypothalamic PVN. We have observed that blockade of opioid receptors reverses the moxibustion blood pressure lowering effect suggesting that the action of moxibustion, in part, likely is processed in this brain region. Thus, temperature-dependent moxibustion at specific acupoint reduces elevated blood pressure through hypothalamic opioid receptors in the PVN and, unlike cardiovascular EA-inhibition, peripheral local TRPV1 receptors.

Point specific stimulation with moxibustion or EA differentially inhibits elevated blood pressure. Current study shows that stimulation at ST36 acupoint with moxibustion is effective in reducing elevated blood pressure in contrast to moxibustion application at G39. In line with these observations, moxibustion at different acupoints induces facilitatory and inhibitory effects on gastric motility (Su et al., 2015) supporting the point specific effect of moxibustion. In addition, stimulation with EA at P5-6 or ST36-37 acupoints inhibits sympathoexcitatory blood pressure responses (Tjen-A-Looi et al., 2004; Zhou et al., 2005a) while current data show the inability of EA-inhibition at G37-39. EA modulates also reflex hypotension and bradycardia with point specific actions (Tjen-A-Looi et al., 2018) suggesting that EA influences both cardiovascular inhibitory and excitatory reflex responses. Collectively, these observations suggest that both moxibustion and EA modify excitatory as well as inhibitory reflex responses by stimulation at specific acupoints.

Transient receptor potential vanilloid 1, a known capsaicin receptor, is heat-sensitive and depolarizes neurons at temperatures greater than 42°C. Interestingly, studies have suggested that ruthenium red, the non-competitive antagonist for the capsaicin receptor, abolish the capsaicin but not the heat induced reflex response (Hiura, 2009). The polymodal TRPV1 receptor, sensor of chemical, mechanical and heat stimuli, is expressed most abundantly in small diameter peripheral sensory neurons (Sanchez et al., 2001; Caterina, 2007). The TRPV1 located on sensory neuronal tissue is a ligand-gated, voltage-gated and cationic channel (Voets et al., 2004; Matta and Ahern, 2007). TRPV1 located on sensory fibers is important during 50 Hz EA ST36 on systemic analgesia (Xin et al., 2016). In these respects, current study shows an important role for TRPV1, likely located in the small diameter fibers underneath acupoint ST36, during moxibustion inhibition of pressor responses, however, this receptor does not participate during the inhibitory actions of 2 Hz EA. Notably, MA also modulates sympathoexcitatory cardiovascular reflex responses through peripheral TRPV1 underneath the blood pressure lowering acupoint P6 (Guo et al., 2018). Hence, TRPV1 activated by heat or mechanical stimuli during moxibustion or MA application respectively modulates sympathoexcitatory cardiovascular reflex responses in contrast to EA-inhibition on pressor responses. Further studies are warranted to examine the role of TRPV1 during actions of EA focusing on physiological conditions and stimulating parameters.

The importance of supraspinal regions during effects of moxibustion has been unclear while EA inhibits cardiovascular responses, in part, through hypothalamus, midbrain and medulla. Stimulation of ST36-37 with EA activates hypothalamic arcuate nucleus, modulates brainstem rVLM activity and decreases sympathoexcitatory cardiovascular reflex responses (Tjen-A-Looi et al., 2004; Li et al., 2006). We also have demonstrated that the PVN projecting to rVLM is activated during EA (P5-6) while the present study shows that moxibustion through local TRPV1 at ST36 reduces reflex increases in blood pressure through the hypothalamic PVN. In accordance with the previous and current studies, activation of peripheral TRPV1 at ST36 modifies hypothalamic PVN, PVN-rVLM projection and hence cardiovascular reflex responses. However, current observation indicates that activation of ST36 by EA does not include the activation of the heat sensitive TRPV1. Future studies are needed to determine the peripheral mechanisms during EA activation of ST36 involving central regions such as PVN in modulating the reflex elevation of blood pressure.

The PVN is rich in opioids. In particular, the opioids, enkephalin and β-endorphin, are present in the PVN and participate in regulation of cardiovascular function (Kiss et al., 1984; Lessard and Bachelard, 2002; Bowman et al., 2013). Furthermore, opioids reduce neuronal activity in PVN in rat hypothalamic brain slice preparation (Muehlethaler et al., 1980; Pittman et al., 1980). In intact animal, we show the relevance of PVN opioid receptors during effects of EA at P5-6 (Tjen-A-Looi et al., 2016). Although stimulation with EA at P5-6 decreases the sympathetic activity of cardiovascular neurons in PVN that, in turn, reduces pressor responses through activation of PVN opioid receptors (Tjen-A-Looi et al., 2016), the actions and effects during ST36 stimulation and activation of the local TRPV1 has been unclear. We currently demonstrate a reversal of the moxibustion-inhibition activating temperature specific TRPV1 on sympathetic cardiovascular responses following non-specific blockade of opioid receptors in the PVN. Thus, the present data show that moxibustion inhibition by stimulation of ST36 and activation of peripheral TRPV1 employs the opioid system in the PVN to reduce sympathoexcitatory reflex responses. The specific opioid receptor subtype(s) in the PVN relevant to the moxibustion-inhibition warrants further investigation.

## Perspective and Summary

Our results suggest that thermal dependent moxibustion stimulating ST36 activates TRPV1 in peripheral sensory nerves, reduces PVN neuronal activity through the opioid system, and decreases sympathoexcitatory cardiovascular reflex responses. Decrease in these cardiovascular reflex responses by stimulation of acupoint ST36 with EA or moxibustion appears to occur through different peripheral mechanisms. These observations imply that the activation of sensory neuron during acupoint stimulation by different modes such as EA, MA, or moxibustion eventually decreases sympathoexcitatory responses possibly through similar central processes (Tjen-A-Looi et al., 2016; Guo et al., 2018). Although previous reports show moxibustion blood pressure lowering effect in combination with antihypertensive drugs, present data show that moxibustion alone decreases sympathoexcitatory blood pressure responses. Studies are warranted to examine the long lasting effect of moxibustion on sustained hypertension.

## Author Contributions

ST-A-L, LC, and PL were responsible for experimental design and data evaluation. The experiments were conducted by ST-A-L, YG, Z-LG, and YP. All authors reviewed the manuscript.

## Conflict of Interest Statement

The authors declare that the research was conducted in the absence of any commercial or financial relationships that could be construed as a potential conflict of interest.
